This article has been retracted.

# Influence of Comprehensive Nursing Intervention Combined with WeChat Platform Propaganda and Education of ERAS Concept on Postoperative Functional Recovery of Patients with Gallbladder Polyps

**DOI:** 10.1155/2022/6919130

**Published:** 2022-08-10

**Authors:** Yan Zhang, Dongmei Guo, Xiaocui Yang, Xiaojing Sun, Yajuan Dong, Jun Zhang, Yujiao Gao, Zhanhua Guo, Haikun Zhou, Quanfu Li

**Affiliations:** Department of Hepatobiliary Surgery, Second Hospital of Baoding, Baoding, Hebei 071051, China

## Abstract

To analyze the effect of comprehensive nursing intervention based on ERAS's concept in laparoscopic gallbladder polyp (GP) surgery on patients' postoperative quality of life and nursing job satisfaction. Ninety patients with polyps were included in this article until October 2021. In this format, the 45 cases are divided into governing bodies and committees according to their processing time. As recommended by the ERAS committee, the committee provides daily and patient care, as well as training on the WeChat platform. The pain level (visual analogue scale (VAS) score), the quality of life (life quality index (GLQI) score), and the incidence of complications were compared between the two groups before and after the intervention. The VAS score of the control group at 2 h after operation was lower than that of the control group, and the difference was statistically significant (*P* < 0.05). After the intervention, the GLQI scores of the two groups were higher than those before the intervention, and the GLQI scores of the control group were higher than those of the control group, with significant differences (all *P* < 0.05). Studies have shown that comprehensive nursing intervention applied to patients with gallbladder polyps can reduce postoperative pain with less complications and can also improve nursing satisfaction, which is worthy of clinical promotion.

## 1. Introduction

ERAS, minimally invasive surgery, and artificial intelligence are three important development directions of modern surgical technology in the twenty-first century. ERAS is not a new surgical technique, but a new concept of perioperative management, which is an important supplement to traditional surgery. ERAS's core principle is to reduce the risk of complications through a multimodal approach to surgical stress response. ERAS operating mode is multidisciplinary collaboration (MDT). This includes disciplines such as surgical anesthesia care, surgical care, nutrition, psychological rehabilitation, and cooperation between patients and their relatives, which are the prerequisites for ERAS. The importance of active participation of patients and their relatives must be emphasized here; otherwise, the effects of ERAS cannot be fully realized [1]. The interdisciplinary optimized perioperative management measures and operation of the MDT process reengineering commonly used measures include preoperative education, preoperative assessment, prevention of complications, shortening the time of fasting before operation, encouragement of the use of minimally invasive surgery, short-acting general anesthesia, local anesthesia multimode analgesia, trying not to place drainage, early postoperative oral feeding, early ambulation, and early catheter removal. Each optimization measure should be supported by evidence-based medical evidence, and perioperative MDT combination should be applied to the same patient in preoperative, intraoperative, and postoperative management. Close collaboration is maintained throughout to achieve the best results, to reduce pain and risk, and to achieve rapid recovery, as shown in Figure 1. ERAS can reduce the stress response, reduce the incidence of surgical complications, and reduce the risk of surgery by improving the conventional treatment process effectively and reasonably. In this way, the postoperative recovery of patients can be accelerated, the postoperative hospital stay can be shortened, the cost of hospitalization can be reduced, the quality of life of patients can be improved, the surgical experience can be improved, and satisfaction can be improved [2]. ERAS's core is to minimize the stress response of the body during the operation and block the conduction of afferent nerve to the stress signal, so as to reduce the psychological and physical damage of patients. Anesthesia management is an important part of ERAS, and the Postanesthesia Care Unit (PACU) is an important part of ERAS anesthesia management. It is aimed at providing regular care to the patient after anesthesia, reducing the incidence of postoperative complications, and improving the quality of anesthesia healing, which is important for the rapid recovery of postoperative patients. Gallbladder polyp, also known as cystic mucosal eminence, is a growth in the gallbladder, including cholesterol polyps, inflammatory polyps, and gallbladder adenomatous polyps, which will increase the risk of cancer if not treated in a timely and effective manner [3]. Clinical surgery is often used to treat gallbladder polyps, but, if the postoperative lack of corresponding nursing guidance, will cause slow recovery of patients and reduced quality of life. Now, for young adults in interpersonal communication more dependent on the online world, WeChat platform is a powerful interactive information communication platform and not only has the function of text; you can also add images, voice, and video, through health preach. WeChat platform could give patients and their families more directly and more rapid and effective nursing knowledge of disease. It not only saves human resources but also enables patients to continue to obtain relevant knowledge after discharge and communicate with medical staff anytime and anywhere, which is an efficient way of working.

## 2. Literature Review

Erman et al. said that in their clinical work, we often see patients with adhesive ileus after abdominal surgery. This has a certain impact on the recovery of patients, to our nursing work caused a certain degree of difficulty [4]. Teo et al. believe that among the many causes of adhesive ileus, the probability of surgical causes is higher. For surgical nursing managers, how to improve perioperative patient management and prevent complications is the key problem that we need to solve and think about [5]. Khojamli et al. believe that the concept of accelerated rehabilitation surgery (ERAS) is a set of optimized interventions based on evidence-based medicine for perioperative management to achieve rapid recovery [6]. Thompson and Haddad said that in order to prevent and reduce postoperative complications in patients undergoing abdominal surgery, promote the early recovery of gastrointestinal function, and achieve rapid recovery of patients, ERAS concept and comprehensive nursing interventions were adopted in the study, which significantly improved the recovery effect of intestinal peristalsis, reduced the incidence of complications, and improved patient satisfaction [7]. Gleadhill et al. said that gallbladder polyp is a common clinical disease. Although it is a benign disease, if not treated in time, it has a certain risk of deterioration. Therefore, surgery should be taken as soon as possible after diagnosis to remove polyps to ensure patient safety [8]. Zer and Kurt believed that in the past, due to the underdeveloped medical technology, gallbladder polyp surgery often brought great trauma and pain to patients, but in recent years, with the continuous development of minimally invasive technology, its application in gallbladder polyp surgery has effectively improved many defects of traditional surgery [9]. Yin et al. believe that, now, more and more patients with gallbladder polyp choose minimally invasive gallbladder polyp removal for treatment, which not only has less trauma, less pain, and lower risk but also has faster postoperative recovery and fewer complications [10]. Gautam et al. thought that surgical treatment alone is not enough to guarantee the prognosis of patients, and the role of nursing intervention is equally important. Only effective nursing intervention in perioperative period can ensure the smooth implementation of surgery and postoperative rehabilitation effect of patients [11]. Boz et al. thought that in the past, routine nursing intervention was generally carried out for patients in the perioperative period, but there are shortcomings of routine nursing intervention, such as the content of nursing is not comprehensive enough, the details of nursing, and the lack of pertinence, which can no longer meet the actual needs of modern clinical nursing work [12]. Wennmacker et al. thought that ERAS's concept combined with comprehensive nursing intervention can change the traditional concept of medical staff and provide comprehensive, systematic, meticulous, and patient nursing services for patients, enabling remarkable recovery effects of intestinal peristalsis. The time to get out of bed and exhaust was shortened significantly, the incidence of adhesive ileus was significantly reduced, and the patients fully mastered the health education content, so that the satisfaction of nursing work will be significantly improved, which is worthy of continuous promotion and application in clinical work [13].

## 3. Method

### 3.1. Research Data

A total of 90 patients with gallbladder polyps who underwent surgery in Chinese medicine between October 2019 and October 2021 were selected and divided into a board and a monitoring team, followed by admission time, and 45 patients in each group. There are 21 men and 24 women on the board. Their age is 29-65, the average age (47.12-4.36). Disease classification is 0.8~4 a, mean (2.12 ± 0.54) a. The study involved 27 men and 18 women. The mean age is 30–60 years, and the mean age is (45.35 ± 6.21). Bacteria range from 1 to 4 a, with an average of (2.36 ± 0.62) a. There were no significant differences in the general data between the two groups (total *P* > 0.05). Patients can participate in this study and sign a consent form. The study was approved by the Medical Health Committee [14]. Inclusion criteria: diagnosis of gallbladder polyp requiring surgical treatment. Exclusion criteria: accompanied by severe cognitive impairment or mental illness; with other serious organic diseases of the whole body.

### 3.2. Nursing Methods

#### 3.2.1. Control Group

Routine care was taken to keep the ward clean and tidy, disinfection was performed once a day, humidity was 50%-60%, and temperature was 24-36°C. Instruct patients to take medicine on time and give routine psychological nursing and diet intervention. Health education was given to patients and their families, including common knowledge of diseases and possible complications, and discharge manuals were issued before discharge [15].

#### 3.2.2. Observation Group

Comprehensive nursing intervention combined with ERAS concept is implemented as follows:

1. Training and testing

Due to the influence of traditional beliefs among health care professionals, there is insufficient awareness of the best evidence for early activity. The department strengthened training and assessment, including abdominal nursing content, the effect of early activities, specific methods, and patient communication skills. The assessment results were included in the department performance assessment, and the training rate and awareness rate reached 100%.

(2) Psychological counseling intervention

Patients and their families think that patients need to recuperate after surgery; nurses should be patient psychological counseling, so that patients will fully remove ideological concerns and active with sports rehabilitation nursing. In ordinary work, we should learn to listen to patients' ideas and perspective-taking, respect patients, to establish a good nurse-patient relationship, and use their own professional knowledge to provide help for patients, so that patients can actively realize the necessity and importance of early postoperative activities.

(3) Dietary intervention

① Eat a soft and digestible diet for lunch before surgery; have a semiliquid diet for dinner, fasting after 00:00, and no drinking after 04:00; ② postoperative dietary intervention according to the site and method of operation to formulate the feeding plan.

(4) Oral intervention

After the operation, prepare a transparent lipstick to apply lips or cucumber slices to apply lips, remember not to use cotton swabs with water to apply lips, air evaporation is easy to dry lips. Prepare a bottle of sugar-free gum (such as patients without dentures under the supervision of family members, the first day after the operation, chew a piece of gum for 10 minutes in the morning and afternoon and spit it out for 7 consecutive days), promote the recovery of intestinal peristalsis, stimulate the increase of saliva secretion, and reduce dry mouth and bad breath.

(5) Abdominal massage

The first day after the operation began to massage along the umbilical circumference, the technique is standard, light, and moderate, two times a day alternately counterclockwise massage, 20 minutes each time, last for a week.

(6) Exercise intervention

After the patient wakes up from anesthesia, raise the head of the bed 30-45 to help the patient turn over. The patient was instructed to exercise in bed on the first postoperative day: ① ankle pump movement: instruct client to lie flat or half-lying→legs straight and together→press the instep so that the toe is as straight as possible (hold 5 s)→return your feet to their original position and swing them to the left (hold 5 seconds)→swing your feet to the right (hold 5 seconds)→return your feet to their original position and rotate clockwise for the maximum possible time→rotate your feet counterclockwise as much as possible→repeat 10 times; this can promote lower limb blood circulation and prevent lower limb venous thrombosis. ② Carry buttock movement: instruct client to lie flat on the bed→apply pressure to the wound from both sides of the waist to prevent pain→step on the bed with your legs bent→lift hips with leg strength (hold 5 s)→gently put your hips back on the bed→repeat the procedure 10 times to promote gastrointestinal motility and help ventilation. ③ Cough movement: instruct client to be in semilying or sitting position→apply pressure to the wound from both sides of the waist to prevent pain→take several deep and slow breaths, then take a deep breath through your nose and hold your breath for 3 seconds→2-3 short, strong deep coughs from the chest, and when sputum is present, cough up the sputum→repeat the procedure 10 more times to help your lungs expand and prevent infection. On the second day after the operation, on the basis of completing the activity goals of the first day, the patients were instructed to sit, sit, stand, and go to the toilet in the ward three times a day for 20-30 minutes each time. Gradually increase the amount and time of activity each day according to the patient's physical fitness and self-perception. In the process of exercise to observe the patient's situation, such as the patient self-feeling palpitation, complexion change sweating, immediately stop the activity, and standardized disposal [16].

(7) Progress of activity

Nursing staff should carefully observe the patient's activity and keep relevant records. For the first time, all activities are encouraged by a nurse at the bedside. Based on the concept of integrated nursing intervention combined with ERAS ERAS, health education via WeChat is established to enable patients and their families to follow the WeChat platform by scanning the QR code, and the nurses in charge will introduce the use of the WeChat platform to patients and their families. The content of WeChat platform mainly includes basic knowledge of diseases (manifestations and treatment process of diseases, etc.), hospital examination (examination items and cost-related to diseases), nursing knowledge (key points of continuing care of diseases, manifestation, and treatment of common complications), and discharge propaganda and education (matters needing attention after discharge, etc.). For patients with gallbladder polyp, postoperative nursing knowledge should be regularly pushed in the continuing care, including the intake of protein and the amount of oxalate-rich food. Pictures and videos of routine gallbladder disease prevention were sent, and a special person was responsible for answering patients' questions on WeChat platform, and a total of 1 month of nursing intervention [17].

### 3.3. Observation Target

Performance-related measures and positive life scores before and after the intervention were evaluated and compared between the two groups.

### 3.4. Statistical Analysis

Statistical software SPSS21.0 was used for data analysis. Measurement data were represented by mean ± standard deviation, $\bar{x}\pm s$, and comparison between the two groups was performed by *t* test. Data collection *x*^2^ was used to compare the groups, and *P* < 0.05 was considered significant.

## 4. Results and Discussion

### 4.1. Operation-Related Indicators

Comparison of surgery-related indicators between the two groups showed that the observation group was significantly better (*P* < 0.05), as shown in Table 1.

### 4.2. Quality of Life Scores before and after Intervention

There was no significant difference in mean life expectancy scores between the two groups prior to the intervention (*P* > 0.05). After the intervention, the control group was as high as shown in Table 2 (*P* < 0.05).

### 4.3. The Degree of Pain 2 H after Surgery

2 h after surgery, VAS score of the observation group (2.96 1.02) was lower than that of the control group (4.88 1.36); the difference was statistically significant (*P* < 0.05).

### 4.4. Incidence of Complications

In the control group, there were 1 case of abdominal bleeding, 3 cases of incision infection, 2 cases of biliary leakage, and 2 cases of biliary duct injury. The complication rate was 19.05%. There was 1 case of biliary duct injury in the observation group, and the complication rate was 2.38%. The control group problems were smaller than those in the control group and differed significantly (*P* < 0.05).

### 4.5. Living Quality

Prior to the intervention, there was no significant difference in GLQI scores between the two groups (*P* > 0.05). After the intervention, the CLQI scores of the two groups were significantly higher than before the intervention, and the control group's GLQI scores were significantly different from those of the control group (both *P* < 0.05), as shown in Table 3.

The interest rates in both groups were 97.23% higher in the control group than in the control group (*P* < 0.05), as shown in Table 4 and Figure 2.

### 4.6. Discussion

ERAS is an important development and revolution in surgery in this century. It is not a single measure, but the integration of a series of optimized measures with the best evidence. The ERAS concept and ERAS care has been widely recognized by the medical community today, and its clinical implementation has been effectively verified [18]. ERAS is also known as accelerated rehabilitation surgery. Traditionally, recovery begins after surgery, so there are many literatures on postoperative care under ERAS's concept, while less attention has been paid to accelerated rehabilitation care during surgery. Surgical patients need a holistic and continuous nursing process, and many factors in the surgical process have been proven to affect patient prognosis. Therefore, nursing management to accelerate the recovery of patients should be advanced to the preoperative and cover the whole operation process. Clinical perioperative management under the current ERAS concept needs to be optimized from the preoperative, intraoperative, and postoperative stages to minimize emergency response and promote recovery. It requires the cooperation of surgeons, anesthesiologists, operating room specialists, nurses, and ward nurses. The development of the ERAS concept to today is no longer to discuss whether it is better than the traditional model, but the implementation and implementation of the concept and strategy. In particular, the application of accelerated intraoperative rehabilitation nursing in patients with gallbladder polyps under ERAS's concept is still in its infancy, requiring a group led by operating room nurses to explore and study the implementation methods of relevant strategies [19]. Through improving the preoperative visit model, scientific management of the preoperative fasting time, optimization of intraoperative temperature management, prevention of intraoperative thrombosis, and improvement of postoperative resuscitation care, ERAS concepts are combined with clinical practice. Starting from the three stages of preoperative, intraoperative, and postoperative surgery, the adverse reactions caused by surgical stress should be minimized, and the tolerance and coping level of surgical patients should be improved as a whole, to improve prognosis and promote rehabilitation. Therefore, the application of accelerated rehabilitation nursing interventions in surgery under ERAS's concept should be studied. It not only enables continuous perioperative holistic nursing concept of ERAS but also has urgent practical significance for further optimizing and standardizing the implementation of relevant strategies of ERAS and also provides scientific theoretical and practical basis for specialized nurses in the operating room to effectively carry out intraoperative accelerated rehabilitation nursing intervention under ERAS concept. Under this ERAS concept, accelerate rehabilitation nursing to reduce operation and stress as the core goal, from optimization of preoperative supervision mode, to ban the scientific management of fasting time, intraoperative blood clots to intraoperative temperature management of prevention, and management optimization to improve postoperative recovery nursing way; notting is not to reduce the operation as the core of the best stress cycle on the basis of clinical practice. Integrated visits to operating rooms and wards reduced preoperative anxiety levels. Stable core body temperature can promote drug metabolism, shorten the recovery time, reduce the incidence of postoperative SSI, and promote postoperative ALT AST recovery. The family arousal pattern reduced the occurrence of EA, improved the quality of resuscitation, and reduced the use of muscle relaxation antagonists for resuscitation and symptomatic treatment of EA. Reduce PACU stay and monitoring time, so that the drug expenditure and PACU monitoring costs will greatly reduce. The reduction of postoperative complications also greatly reduces the cost of subsequent treatment. The relative stability of the patient's internal environment and the improvement of the overall tolerance to surgery can promote rehabilitation without compromising the safety of the patient's treatment, thus shortening the length of hospitalization and reducing hospitalization costs [20]. This makes intraoperative care under the ERAS concept cost-effective in many aspects of clinical practice. Traditional health knowledge propaganda adopts oral education or paper version of the propaganda, one is not wide enough, and two is lack of vitality; the content is monotonous and boring. The health promotion on WeChat, the most widely used social network platform, is making up for these shortcomings. You can receive text, pictures, voice, and video messages with your mobile phone. Compared with traditional health education, WeChat platform is more specific, more convenient, and vivid. Not only patients but also the public can learn relevant knowledge about diseases anytime and anywhere. Meanwhile, it can also stimulate the public's initiative to explore more medical health knowledge, which effectively improves the effect of health education [21]. WeChat platform use is not restricted by time and space, can arrange one or more according to the needs of clinical medical personnel to handle, not only save human resources, and improve the patient's satisfaction, to improve the quality of life of patients after discharge and the lack of medical professional knowledge of patients, and their families do not have to bother to identify the authenticity of information. Through WeChat platform, the hospital can receive timely feedback from patients and urge patients to come to the hospital for regular review. Medical staff can help discharged patients deal with problems in a timely manner, which not only makes patients feel relieved but also enables medical staff to accumulate more relevant knowledge and experience [22]. In addition, the results of this study showed that after different propaganda and education methods in continuous care, patients in the observation group had a deeper understanding of the disease than those in the control group and were more satisfied with the health propaganda and education methods on WeChat platform.

## 5. Conclusion

Gallbladder polyp is a common gallbladder disease. The common symptoms are abdominal bloating, nausea, and vomiting. If not treated in time and effectively, it can be developed into gallbladder cancer. Common surgical treatment has many risks such as improper surgical stress response and nursing, leading to a high incidence of postoperative complications and delaying the rehabilitation process. Therefore, should be in the treatment at the same time should cooperate with scientific and effective nursing intervention measures; comprehensive nursing intervention emphasizes in the preoperative, intraoperative, and postoperative stages according to the patient's physiological, psychological, cultural, and spiritual needs in many aspects, to provide the best way of nursing. Before surgery, health education and psychological counseling were carried out to prepare for surgery, relieve tension and anxiety, improve patient compliance, and enhance confidence. During the operation, we strictly followed the operation procedures, paid close attention to the changes of patients' vital signs, and timely dealt with the abnormal conditions. After surgery, we conducted intervention on patients' postural activities, abdominal drainage, lifestyle, diet, etc. The results of this study showed that VAS score and complication rate of the observation group were lower than those of the control group after intervention, indicating that this nursing mode can relieve pain and reduce complications. In this study, through preaching during hospitalization, patients were improved to be familiar with the knowledge of disease etiology care and treatment, to enhance their confidence in recovery, to guide reasonable diet, regular life, appropriate exercise, work, and rest, and to avoid mental tension or overwork. GLQI scores in both groups after intervention were higher than before intervention, and GLQI scores in the control group were higher in the control group, indicating that health care can improve the quality of care, improving postoperative well-being of patients with gallbladder polyps. In conclusion, good health care reduces pain and discomfort in patients with gallbladder polyps and improves quality of life. They were divided into control groups and controlled groups using a sequential distribution procedure, with 45 patients in each group. The board provided regular caregivers and the care team provided health information on WeChat as part of routine care. To sum up, WeChat integrates functions such as text, voice, pictures, and video, which makes it easier for the public to accept and understand and has the advantages of economy, simplicity, and effectiveness. Health education based on WeChat platform can significantly improve patients' satisfaction and awareness of the disease and is more conducive to patients' health recovery in continuous care. Health education on WeChat platform has improved patients' and their families' understanding of disease-related knowledge and stimulated the public's initiative to learn medical knowledge in daily life, which is worthy of further promotion in clinical practice.

## Figures and Tables

**Figure 1:** ERAS concept map.

**Figure 2:** The line chart of nursing job satisfaction was compared between the two groups.

**Table 1:** Comparison table of operation-related indicators between the two groups.

Group	Time to get out of bed (h)	Anus exhausting time (h)	Length of stay (d)
Observation group (*n* = 45)	8.85 ± 1.61	15.32 ± 3.40	4.51 ± 0.88
Control group (*n* = 45)	12.24 ± 1.98	20.33 ± 4.14	6.21 ± 1.02
*t*	8.351	5.928	8.705
*P*	<0.05	<0.05	<0.05

**Table 2:** Comparison of quality scores of the two groups before and after the intervention.

Group	Physical function		Mental functioning	
	Before the intervention	After the intervention	Before the intervention	After the intervention
Observation group (*n* = 29)	56.58 ± 6.99	78.24 ± 6.25	55.15 ± 5.95	8123 ± 6.78
Control group (*n* = 29)	56.43 ± 5.14	66.85 ± 7.21	54.98 ± 5.28	70.27 ± 6.98
*t*	0.026	7.182	0.028	8.147
*P*	> 0.05	<0.05	>0.05	<0.05

**Table 3:** Comparison of GLQI scores between the two groups before and after intervention.

Group	Number of cases	GLQI score	
		Preoperative	Postoperation
Control group	45	81.65 ± 14.95	94.51 ± 17.95
Observation group	45	80.35 ± 15.24	108.26 ± 20.65

**Table 4:** Nursing job satisfaction was compared between the two groups.

Group	Number of cases	Great satisfaction	Satisfaction	Dissatisfaction	Nursing job satisfaction
Observation group	45	29	16	0	45 (100%)
Control group	45	27	11	7	38 (84.44%)
*x* ^2^					8.347
*P*					0.004

## Data Availability

The data used to support the findings of this study are available from the corresponding author upon request.
